The article "Modeling Brain Somatic Mosaicism With Cerebral Organoids, Including a Note on Mutant Microglia" was retracted in 2020. Reasons: no approval from the institution; no approval from a third party; copyright claims; concerns about the citations.

# Modeling Brain Somatic Mosaicism With Cerebral Organoids, Including a Note on Mutant Microglia

**DOI:** 10.3389/fnmol.2019.00277

**Published:** 2019-11-14

**Authors:** Bert M. Verheijen

**Affiliations:** ^1^Department of Translational Neuroscience, UMC Utrecht Brain Center, University Medical Center Utrecht, Utrecht University, Utrecht, Netherlands; ^2^Department of Neurology and Neurosurgery, UMC Utrecht Brain Center, University Medical Center Utrecht, Utrecht University, Utrecht, Netherlands

**Keywords:** brain genomic mosaicism, somatic mutations, neurogenetics, induced pluripotent stem cells, cell models, 3D organoids, neural circuits, neurological disorders

## Abstract

The brain is a genomic mosaic. Cell-to-cell genomic differences, which are the result of somatic mutations during development and aging, contribute to cellular diversity in the nervous system. This genomic diversity has important implications for nervous system development, function, and disease. Brain somatic mosaicism might contribute to individualized behavioral phenotypes and has been associated with several neuropsychiatric and neurodegenerative disorders. Therefore, understanding the causes and consequences of somatic mosaicism in neural circuits is of great interest. Recent advances in 3D cell culture technology have provided new means to study human organ development and various human pathologies *in vitro*. Cerebral organoids (“mini-brains”) are pluripotent stem cell-derived 3D culture systems that recapitulate, to some extent, the developmental processes and organization of the developing human brain. Here, I discuss the application of these neural organoids for modeling brain somatic mosaicism in a lab dish. Special emphasis is given to the potential role of microglial mutations in the pathogenesis of neurodegenerative diseases.

## Introduction

Elucidating the architecture of the brain is central to understanding brain function and susceptibility to disease. The brain is highly complex, and progress in understanding the brain will largely depend on the development of new technologies and concepts that allow us to investigate its complexities in detail. Emerging evidence suggests that the human brain can be considered a complex “mosaic” of genetically different cells (Rohrback et al., 2018). This genomic mosaicism is brought about by somatic mutations, i.e., post-zygotic changes to the genome that arise during a lifetime as opposed to being inherited. Brain somatic mosaicism has been linked to several neurodevelopmental disorders (D’Gama and Walsh, 2018; Ye et al., 2019) and may contribute to the etiology of age-related neurodegenerative diseases (Leija-Salazar et al., 2018; Verheijen et al., 2018). Moreover, somatic mutations may be involved in generating cellular diversity in the neurotypical brain (McConnell et al., 2017). Any type of genomic change occurring post-zygotically [e.g., indels, CNVs, SNVs, L1 retrotransposition events (Misiak et al., 2019; Zhao et al., 2019), etc.] can contribute to tissue mutational mosaicism, and, although most somatic mutations are presumably silent (e.g., synonymous, non-coding), some of these can affect gene expression, cell survival, and neural circuit performance, thereby influencing functional heterogeneity. For example, select mutations (driver mutations) could impact cellular fitness and confer clonal competitive advantage or disadvantage during development. Interestingly, CNV neuron frequency was found to be anti-correlated with age in human brain, indicating that many CNV neurons are selectively vulnerable to aging-associated atrophy (Chronister et al., 2019).

The article "Modeling Brain Somatic Mosaicism With Cerebral Organoids, Including a Note on Mutant Microglia" was retracted in 2020. Reasons: no approval from the institution; no approval from a third party; copyright claims; concerns about the citations.

Despite their potential significance to brain function and disease, the precise origins and consequences of specific brain somatic mutations remain largely unclear. Analysis of human post-mortem tissue specimens, while important, only provides a snapshot of what is occurring in the brain. In order to study brain somatic mosaicism in detail, it will be necessary to use models. In this, choosing the right experimental system to answer the questions at hand will be critical: a model has to be complex enough to recapitulate sufficient aspects of brain mosaicism, yet simple enough to study in depth.

Cerebral organoids, generated from human induced pluripotent stem cells (hiPSCs), have emerged as three-dimensional (3D) models of the human brain, mimicking various features of the developing brain at the cellular, molecular, and electrophysiological level (Lancaster et al., 2013; Lancaster and Knoblich, 2014; Di Lullo and Kriegstein, 2017; Amin and Paşca, 2018; Paşca, 2018; Giandomenico et al., 2019; Kanton et al., 2019; Trujillo et al., 2019; Yakoub, 2019). In combination with techniques to probe and manipulate tissues, such as single-cell genomics and genome editing technologies, these organoids can bring unprecedented insight into human brain development and various human brain pathologies. Here, the use of cerebral organoids as models for brain somatic mosaicism is discussed. Special attention is given to the possible role of microglial mutations in neurodegenerative disease.

## Somatic Mosaicism in Cerebral Organoids

Somatic mutations occur at various time points during development and aging (Figures 1A–C), yet the functional implications of somatic mutations in the nervous system remain largely unknown. *De novo* somatic mutations have been traditionally studied in cancer, but not in normal cells. To study brain somatic mosaicism in detail, it is imperative to use models. I suggest that hiPSC models, including cerebral organoids, are especially attractive systems to elucidate underlying mechanisms. Cerebral organoids are microscopic self-organizing, 3D structures that are grown from stem cells *in vitro* and recapitulate several structural and functional aspects of the developing brain (Lancaster et al., 2013). 3D neuronal differentiation has already been combined with CRISPR/Cas9 genome editing to investigate the “two−hit” hypothesis of cortical tuber development (a model involving second-hit somatic mutations) in human cortical spheroids (Blair et al., 2018). Additionally, cerebral organoids have been used as models for tumorigenesis using CRISPR/Cas9 oncogene manipulation (Bian et al., 2018; Ogawa et al., 2018).

The article "Modeling Brain Somatic Mosaicism With Cerebral Organoids, Including a Note on Mutant Microglia" was retracted in 2020. Reasons: no approval from the institution; no approval from a third party; copyright claims; concerns about the citations.

**FIGURE 1:** Modeling brain somatic mosaicism in cerebral organoids. **(A)** From zygote (Z) to birth and after, somatic mutations occur in the genomes of cells. These mutations result in somatic mosaicism, i.e., the presence of genetically distinct populations of cells within an individual. Normal tissues, including the brain, are mosaics of clones of various sizes wherein each cell’s genome is unique. Through genome sequencing, somatic mutations can actually be used to trace complete cell lineage trees (Behjati, 2016; McKenna and Gagnon, 2019). The mutation rate μ (probability of a mutation occurring per cell division) equals the number of mutation events (*v*) divided by the number of cell divisions (*D*). In the example μ = 1/7 mutations per genome per cell division. The mutation frequency *f* (proportion of mutant cells in a population) is the number of mutant cells in a population (*M*) divided by the total number of cells in a population (*N*). In the example *f* = 2/8. **(B)** Somatic mutations occur throughout development and aging. Mutations in early development can affect a large number of cells and will be shared among various tissues (green triangle). Mutations occurring later in development will be limited to a smaller number of cells (blue triangle), e.g., brain-specific mutations. Mutations occurring in post-mitotic cells result in very fine changes, as these are confined to single cells (red triangle). The estimated average mutation rate during neurogenesis (∼5.1 SNVs per day per progenitor, corresponding to ∼8.6 SNVs per division per progenitor) has been found to be higher than the mutation rate during early embryogenesis (∼1.3 SNVs per division per cell) (Bae et al., 2018). From an evolutionary point of view, this ramping up of mutation rate during neurogenesis is not very surprising. After all, protecting the genome at early embryonic stages is more important than at later stages of differentiation, where these mutations will affect fewer cells. Postnatally, after the rapid cellular expansion that happens during development, the mutation rate slows down considerably. **(C)** Somatic mutations continue to accumulate over a lifetime. It has been suggested that accumulation of mutations could cause aging (Failla, 1958; Szilard, 1959), but this remains to be proven (Niedernhofer et al., 2018; Zhang and Vijg, 2018). Recent data support a model wherein mutations accumulate age-dependently in single neurons (Lodato et al., 2018), and it was proposed that age-related accumulation of mutations in a diploid genome could provide a model for the exponential occurrence of age-related disease (following Gompertz kinetics). Most genes can function with one remaining allele, so for many years single mutations would have little effect on gene function (although a lot of genes are dosage-sensitive). During aging, mutations would then increasingly knockout the remaining allele or genes, creating “zombie cells” that are complete knockouts for essential genes. In neurodegenerative diseases like AD, oxidative stress and DNA damage are increased, making it likely that somatic mutation burden is increased in affected neurons. **(D–F)** Various approaches can be devised to model somatic mosaicism in cerebral organoids, including: generating cerebral organoids from mixed cultures of genetically different hiPSCs **(D)**, transfection of cerebral organoids with gene-editing constructs **(E)**, or combining genetically different hiPSC-derived cells into fused cerebral organoids **(F)**. **(G)** Mosaic cerebral organoids can be analyzed by multiple methods, such as single-cell sequencing, proteomics, epigenetic analysis, live imaging, tissue clearing and 3D reconstruction, optogenetic probing, and electrophysiology (e.g., patch-clamping or multi-electrode recordings) (Amin and Paşca, 2018). Xenotransplantation of the organoids to mouse brains can be considered to study *in vivo* effects (Mansour et al., 2018). Cerebral organoids can also be used for pharmacological testing.

The article "Modeling Brain Somatic Mosaicism With Cerebral Organoids, Including a Note on Mutant Microglia" was retracted in 2020. Reasons: no approval from the institution; no approval from a third party; copyright claims; concerns about the citations.

Multiple methods to accomplish genomic mosaicism in cerebral organoids are proposed:

(1) *Mixing*. Co-culture of hiPSC cells with different genotypes is a straightforward strategy to generate mosaics (Figure 1D). In this approach, isogenic pairs of gene-edited and control hiPSCs could be cultured together to make mixed cerebral organoids. The resulting organoids can then be used to understand how genetic variation gives rise to variation in cellular phenotypes. A potential problem of this approach, however, is maintaining cellular diversity in culture. Variation in cellular growth rates and somatic selection could be part of a mosaic phenotype, but for many downstream analyses, stable organoids that include a fraction of cells derived from all donor hiPSC populations are required. Using different ratios of donor cells for cerebral organoid differentiation could solve this problem. Additionally, mutations that confer selective advantage could be acquired in culture (Merkle et al., 2017). Careful genome-wide analyses will be necessary to prevent phenotypes that arise due to acquired mutations. An interesting addition to this co-culture method would be the incorporation of inducible donor hiPSCs, allowing for induction of mutant cells at a later time point, e.g., by adding Cre recombinase to the organoid.

(2) *Transfection*. Local genome editing in cerebral organoids could be achieved by transfection of CRISPR/Cas9 constructs (Figure 1E). In mouse brain, single cells can be transfected by *in utero* electroporation to generate mosaics for functional analysis (McConnell et al., 2017). Similarly, gene-editing plasmids can be injected into cerebral organoids (e.g., into the ventricle-like, fluid-filled cavities) and electroporated into surrounding cells (Lancaster et al., 2013). Alternative strategies, such as viral vector-based delivery of CRISPR/Cas9, can also be considered to successfully attain genome editing in organoids.

(3) *Fusion*. Different brain organoids can be fused to generate “assembloids” that model brain regional interconnectivity (Birey et al., 2017). Combining gene-edited and control cerebral organoids for organoid fusion would result in brain assembloids of genetically different cells (Figure 1F). Interestingly, cerebral organoids have also been combined with other, non-neuronal cell types, e.g., microglia-like cells, to model neuro-immune interactions (Abud et al., 2017; Lin et al., 2018). In another study, cerebral organoids were combined with patient-derived glioblastoma cells and organoid-derived tumor cells to model tumor growth (Ogawa et al., 2018). These approaches could also be used in the context of brain somatic mosaicism, to introduce mutant cells into control cerebral organoids or vice versa.

Choosing the best approach for studying brain somatic mosaicism will depend on the specific questions being asked and on technical considerations. For example, local transfection of genetically defined cerebral organoids could be a good strategy to introduce second-hit somatic mutations as a model for focal cortical dysplasias, but mixing may be a better strategy for modeling clonal somatic selection during early brain development.

The article "Modeling Brain Somatic Mosaicism With Cerebral Organoids, Including a Note on Mutant Microglia" was retracted in 2020. Reasons: no approval from the institution; no approval from a third party; copyright claims; concerns about the citations.

Mosaic cerebral organoid models can eventually be used for multiple downstream analyses. Examples include (single-cell) sequencing, live imaging, and electrophysiology analysis (Amin and Paşca, 2018; Paşca, 2018) (Figure 1G). Combining different types of analyses will undoubtedly contribute to a better understanding of the functional implications of brain somatic mosaicism.

## Somatic Mutations in Microglia

Somatic mutations could also affect non-neuronal cells, such as neuroglia, which roughly equal the number of neurons in human brain (von Bartheld et al., 2016). For example, it has been demonstrated that introducing oncogenic mutations in the *Braf* gene (RAS/MEK/ERK pathway) in microglial precursors leads to a severe late-onset neurodegenerative disorder in mice (Mass et al., 2017). Mosaic mutant mouse microglia display an activated phenotype and are found in areas with neuronal loss, demyelination, and deposits of amyloid precursor protein (APP). Analysis of brain tissue samples from patients with histiocytic disorder-associated neurodegenerative disease who carried a *BRAF* mutation confirmed that this mouse model recapitulates hallmark features observed in corresponding human pathology (Mass et al., 2017).

Mouse microglia appear to be somewhat different from human microglia, showing species-specific patterns of gene expression and differences in response to aging (Galatro et al., 2017; Gosselin et al., 2017), and it would be interesting to test whether mutations in human microglia produce similar phenotypes experimentally. hiPSC-derived models, like cerebral organoids, could be utilized to investigate this further. Cerebral organoids are generally assumed to be devoid of microglia, due to the non-neuroectodermal developmental origin of these cells. *In vivo*, microglia predominantly develop from primitive erythro-myeloid progenitors in the extraembryonic yolk sac. These progenitors migrate to and colonize the early embryonic brain, where they differentiate into mature microglia (Ginhoux et al., 2010, 2013; Thion et al., 2018). However, in a recent study, cerebral organoids were reported to contain microglia-like cells that are immunopositive for the microglia marker Iba1 and show typical microglia morphology (Ormel et al., 2018). This is in agreement with our previous findings on microglia-like cells in cerebral organoids (Figures 2A–E and Supplementary File 1; Verheijen et al., unpublished data). In earlier work, mesodermal precursors were identified in cerebral organoids through single-cell sequencing experiments (Quadrato et al., 2017). Thus, despite early patterning to a neuroectodermal fate, brain organoids appear to produce a minority of cells of other embryonic origin. These mesodermal precursors in cerebral organoids can probably differentiate into microglia-like cells: the 3D neural niche in the organoids likely provides a suitable environment for the development of microglia (Gosselin et al., 2017) (Figure 2F). It is currently unclear whether the first microglia-like progenitors that are observed arise within typical cerebral organoids or if they originate from yolk sac-like structures that are present in mixed organoid cultures, invading the cerebral organoid after their genesis.

The article "Modeling Brain Somatic Mosaicism With Cerebral Organoids, Including a Note on Mutant Microglia" was retracted in 2020. Reasons: no approval from the institution; no approval from a third party; copyright claims; concerns about the citations.

**FIGURE 2:** Presence of microglia-like cells in cerebral organoids. **(A)** Schematic diagram of the cerebral organoid protocol. First, human induced pluripotent stem cells (iPSCs) are seeded in microwells to induce embryoid bodies (EBs) (*day 0–6*). EBs are structures that form by spontaneous aggregation of pluripotent stem cells into 3D structures and are used to induce germ layer formation. Next, EBs are transferred to neural induction medium to induce neural ectoderm (*day 6–10*). On *day 11*, neuroectodermal tissues are transferred to droplets of Matrigel. Matrigel resembles the complex extracellular environment found in tissues and promotes neuroepithelial bud expansion. Finally, Matrigel droplets containing expanded neuroepithelium are transferred to a spinning bioreactor, to allow further tissue growth and expansion (*day 15–60*). hES medium, human embryonic stem cell medium; A, vitamin A (retinoic acid). **(B,C)** Staining for microglia (Iba1) reveals multiple immunoreactive cells, scattered throughout cerebral organoids. Iba1-positive cells exhibit ramified morphology and are found in proximity of neuronal processes (Tuj1), hinting at direct interactions with neurons. 40-μm-thick sections cryosections were used for all experiments. Scale bars (B) = 500 μm (C) left panel 100 μm,middle panel 50 μm, right panel 20 μm. **(D)** Iba1-positive cells in cerebral organoids express CD68. Scale bar = 20 μm. **(E)** Quantification of Iba1-positive cells in cerebral organoid sections (*n* = 10) reveals substantial organoid-to-organoid variability and/or intra-organoid heterogeneity. **(F)** Proposed model for the development of mesodermal progenitors into microglia-like cells in cerebral organoids. The organoid neuronal niche provides a suitable environment for survival and development of microglia-like cells, for example by expressing certain cytokines (e.g., CSF1, IL-34, TGFβ). CSF1, colony-stimulating factor 1; IL-34, Interleukin-34; MEF2C, myocyte-specific enhancer factor 2C; SALL1, Sal-like protein 1; TGFβ, transforming growth factor-β.

The article "Modeling Brain Somatic Mosaicism With Cerebral Organoids, Including a Note on Mutant Microglia" was retracted in 2020. Reasons: no approval from the institution; no approval from a third party; copyright claims; concerns about the citations.

The description of microglia-like cells arising within brain organoids may have important implications. Recent advances in stem cell technology have resulted in methods to produce hiPSC-derived microglia-like cells *in vitro* (Muffat et al., 2016; Abud et al., 2017; Pandya et al., 2017) [for an overview, see (Pocock and Piers, 2018)]. It has been suggested that a two-step model, in which hiPSC-microglia are first generated based on ontogeny and then conditioned by a tissue-specific environment, e.g., cerebral organoids, holds great potential for microglia modeling (Lee C.Z.W. et al., 2018). However, if some microglia-like cells also develop endogenously within cerebral organoids, this may complicate such an approach. It is recommended that the occurrence of microglia-like cells in cerebral organoids be thoroughly examined in future experiments. Suppression of alternative (non-neuroectodermal) cell fates and/or stimulation of neuralization, e.g., by dual SMAD inhibition (Chambers et al., 2009), in organoid protocols will probably result in brain organoids with improved purity and reduced variability, contributing to their effective use in disease modeling, drug discovery and personalized medicine.

Incorporating mutant hiPSC-microglia-like cells into well-defined cerebral organoids could be one way to study the effects of mutant microglia *in vitro*. Alternatively, an interesting approach would be to use chimeric mice for studying mutations in human microglia in the context of the living mammalian brain (Hasselmann et al., 2019). It is anticipated that the consequences of brain somatic mutations in non-neuronal cells (not only microglia, but also other cells including astrocytes and oligodendrocytes) are more significant than previously appreciated, challenging the traditional neuron-centric view of neurodegenerative disease.

## Outlook

Brain somatic mosaicism has been associated with several neurodevelopmental, psychiatric, and neurodegenerative disorders (Poduri et al., 2013; D’Gama and Walsh, 2018; Leija-Salazar et al., 2018; Verheijen et al., 2018; Nishioka et al., 2019) and may be pertinent to cellular diversification in neurotypical brains (McConnell et al., 2017). For example, genomic mosaicism could lead to fitness-based cell selection during neural circuit development and may affect neural circuit performance. Developmental mutagenesis might be a mechanism for the regional onset and focal pathology seen in many sporadic neurdegenerative disorders (Frank, 2010; Keogh et al., 2018), and somatic mosaicism could even explain the selective vulnerability of certain neurons to aging and disease (Chronister et al., 2019). Excitingly, a recent study showed that the Alzheimer’s disease (AD)-related gene *APP* undergoes somatic recombination in adult neurons (Lee M.H. et al., 2018), which puts an entirely different complexion on the matter (Box 1).

The article "Modeling Brain Somatic Mosaicism With Cerebral Organoids, Including a Note on Mutant Microglia" was retracted in 2020. Reasons: no approval from the institution; no approval from a third party; copyright claims; concerns about the citations.

**Somatic gene recombination in neurons?**

Early speculations on the basis of neuronal diversity in the brain involved gene recombination (Dreyer et al., 1967), similar to the mechanism of antibody diversification in immune cells that was identified later on (Hozumi and Tonegawa, 1976; Tonegawa, 1983). The detection of genomic mosaicism in brain suggests that neuronal genomes are dynamic and that gene recombination might indeed occur in brain cells (Rohrback et al., 2018). In a recent study, Lee et al. provide compelling experimental evidence for somatic recombination in neurons, involving the AD-related gene *APP* (Lee M.H. et al., 2018). They describe a process that involves transcription influenced by neural activity, DNA strand breaks, reverse transcriptase activity, and age. Mosaic incorporation of *APP* variants by reverse transcription [producing *APP* genomic complementary DNAs (gencDNAs)] potentially results in toxic proteins that contribute to sporadic AD (Lee M.H. et al., 2018). Interestingly, *APP* gencDNA sequences were also identified in an unrelated whole-exome pull-down study (Park et al., 2019). If confirmed by other research groups, these data add a new layer of complexity to AD pathogenesis and potentially to neurobiology in general.

The study by Lee et al. also raises many questions (Lee and Chun, 2019):

(i) Are mutant APP proteins present in human brains? Although it is mentioned that the *APP* variants are translated into proteins, further experimental confirmation in post-mortem AD tissue is needed. It has been demonstrated previously that specific antibodies can be used to detect APP mutant proteins in neurons of AD brains (van Leeuwen et al., 1998). The APP^+1^ mutants described by van Leeuwen et al. (1998) were not detected in the data published by Lee et al., but might have been missed due to limited coverage.
(ii) How do the mutant APP proteins confer toxicity? Which pathways are affected by these mutant APP proteins (e.g., APP processing, intracellular trafficking, protein quality control, synaptic function)? The authors express some mutant APPs in a cell line, but it would be interesting to investigate the effects on human stem cell-derived neurons or in an *in vivo* model. It will be important to incorporate the findings into a relevant model system that preferably also includes other cell types (De Strooper and Karran, 2016). It would be interesting to express these mutant APPs in human cerebral organoids.
(iii) Are these recombination events a cause or consequence of neurodegeneration in AD? If these events occur early in disease, can they provide new clues about AD etiology? Only few AD cases are “familial.” What drives the *APP* recombination? Are there genetic risk factors that mediate the propensity for genomic mosaicism? Are there environmental triggers (e.g., physical trauma, exposure to toxins, infections, early life stress)? Intriguingly, observations in mice indicate that early life experience can drive somatic variation in the genome via L1 retrotransposons (Bedrosian et al., 2018).
(iv) Is *APP* retro-insertion into the genome random or does it occur more frequently in certain genomic regions? What are the precise roles of DNA strand break and repair (Alt and Schwer, 2018)? Does the mechanism involve pathways that are also used by transposable elements?
(v) Does the mechanism apply to other genes and can it be linked to other neurological diseases, e.g., Parkinson’s disease or amyotrophic lateral sclerosis? For example, Lee and colleagues did not find gencDNA variants in Presenilin-1 (*PSEN1*), another gene involved in AD.
(vi) What are the clinical implications of the findings? Can these mutational events serve as biomarkers? If rogue APP variants are key players in AD pathogenesis, could this explain the failure of previous clinical trials in AD (e.g., secretase inhibitor trials)? And could these mutant APPs be targeted, e.g., with reverse transcriptase inhibitors or antisense oligonucleotides directed against the most toxic forms?

The article "Modeling Brain Somatic Mosaicism With Cerebral Organoids, Including a Note on Mutant Microglia" was retracted in 2020. Reasons: no approval from the institution; no approval from a third party; copyright claims; concerns about the citations.

Although their potential impact on brain function and disease is huge, the precise consequences of brain somatic mutations remain largely unclear. In addition to developing better methods to identify and validate somatic mutations in brain cells (McConnell et al., 2017; Dou et al., 2018), it will be crucial to interrogate the functional consequences of brain somatic mutations. hiPSC-based models represent a straightforward means to do this. hiPSCs are human cells that retain genetic information from the (patient) donor, can be differentiated toward relevant neural cell types, and represent a virtually unlimited source of cells for long-term experiments. Cerebral organoids generated from hiPSCs offer unprecedented possibilities to study aspects of human brain development and disease in 3D (Lancaster et al., 2013; Paşca, 2018). In this perspective, it is put forward that cerebral organoids can also be used as models for brain somatic mosaicism. Cerebral organoids have several advantages over other model systems, as they are more physiologically relevant than 2D monolayer cultures and are more amenable to manipulation than *in vivo* models. Multiple approaches can be devised to model brain somatic mosaicism in cerebral organoids, such as mixing of donor cells and local transfection of organoids. It is tempting to speculate that somatic mutations in peripheral tissues (e.g., gut, blood) may also contribute to brain disease, e.g., in Parkinson’s disease, where pathological proteins might spread from gut to brain (Kim et al., 2019), and that mutations in non-neuronal brain cells can result in neurodegenerative changes (Mass et al., 2017). Organoid fusion presents an opportunity to address these questions.

The article "Modeling Brain Somatic Mosaicism With Cerebral Organoids, Including a Note on Mutant Microglia" was retracted in 2020. Reasons: no approval from the institution; no approval from a third party; copyright claims; concerns about the citations.

It is important, however, to keep in mind the limitations of these hiPSC-derived systems (Paşca, 2018; Qian et al., 2019). Brain organoids can recapitulate important aspects of brain development, but established protocols are prone to variable results. Organoid size and morphology can be highly variable, even within a single batch of organoids derived from a single hiPSC donor line. Cellular composition of cerebral organoids can also vary substantially, probably due to the stochastic nature of the differentiation process (Amin and Paşca, 2018). Moreover, aging signatures will be lost with hiPSC approaches, because the hiPSC reprograming acts as a developmental reset (Studer et al., 2015; Mertens et al., 2018). Additionally, inter-laboratory variation in neuronal differentiation from pluripotent stem cells has been described (Volpato et al., 2018), and batch-to-batch variation has also been reported for other types of organoids (Phipson et al., 2019). Pre-patterning protocols and other improvements will likely result in organoid cultures that are more consistent and reliable (Cakir et al., 2019; Qian et al., 2019; Velasco et al., 2019), but achieving a complex and well-structured tissue organization that accurately resembles that of the mature human brain remains a challenge with the current organoid models.

Despite their limitations, it is expected that cerebral organoids, in combination with other *in vitro*, *in silico*, and *in vivo* models, will ultimately contribute to a better understanding of brain somatic mosaicism.

## Data Availability Statement

All datasets generated for this study are included in the article/Supplementary Material.

## Author Contributions

The author confirms being the sole contributor of this work and has approved it for publication.

## Conflict of Interest

The authors declare that the research was conducted in the absence of any commercial or financial relationships that could be construed as a potential conflict of interest.
